# Translation of Japanese Literature Language and Natural Language Environment Understanding Based on Artificial Neural Network

**DOI:** 10.1155/2022/2015763

**Published:** 2022-09-16

**Authors:** Lisha Gu

**Affiliations:** Yancheng Institute of Technology, Yancheng 224051, China

## Abstract

Literary translation encompasses not only the communication of ideas across cultures but also the conversion of one word into another. The translation of Japanese literature will, therefore, undoubtedly convey this foreign culture. This study examines the semantic expression of words, the NN model for common sense reasoning, the method of building a common sense knowledge base, and the translation of Japanese literary language with an emphasis on the semantic expression and reasoning methods of natural language based on NN. The network structure, parameter processing, learning algorithm, and learning samples are all discussed in detail at the same time as the integrated NN model is presented. According to simulation results, this algorithm can achieve an accuracy of about 95% and a recall rate of about 96.5%. In addition to greatly enhancing the model's flexibility and popularity, this approach successfully addresses the issue of information loss. It can offer some references for both the translation of literary language and the understanding of natural language.

## 1. Introduction

As they pursue both a material and a spiritual life, modern people are becoming more and more concerned with the quality of life. Japanese literature is one of the literary works that more and more people are starting to read in this situation [1]. Currently, translation is necessary for the spread of literature; however, due to the requirement for language conversion, translators must pay more attention to different cultures and develop their understanding of Japanese literature in order to further encourage the exchange of cultures. Natural language processing covers a wide range of research topics, and semantic expression of natural language, which aims to solve how to make machines express and understand the semantics of natural language efficiently and reasonably, has always been one of them. The discourse meanings that are communicated by natural language in different linguistic granularities are referred to as semantics in natural language. Tagging tasks include a wide range of common NLP tasks, including named entity recognition, part-of-speech tagging, fast word segmentation, and Chinese word segmentation. These tasks not only have real-world applications but they also have an immediate impact on how well more involved NLP tasks perform. Machine translation (MT) is a significant area of research that combines artificial intelligence and natural language processing [2, 3]. It converts one natural language into another using computer-related operations under the assumption that the original meaning will be preserved, realizing the mutual translation between two natural languages and concluding the equivalent conversion of information between different languages. Because of its quick speed and low cost, MT is regarded as a crucial tool for bridging language barriers. However, MT still has a long way to go and its impact is still very different from that of human translation [4]. The study of neural MT still has a lot of room for improvement at this time. The quality of the translations in the corpus used for traditional neural MT training is uneven, and there are numerous translations of the same term, which also negatively affects the performance of literary language translation. Therefore, the study of ANN (artificial neural network) based on natural language understanding and translation of Japanese literary language has great academic significance.

The two main technical approaches used by MT at the moment are rule-based and template-based. Both of these approaches are essentially rule-based, but the template is an elaborate rule with fewer restrictions. The structure of natural language is complex and flexible in comparison to that of images and speech, so it is necessary to alter the DL (deep learning) model to better handle its complex structure. The original feedforward deep network model of the NN (neural network) [5, 6] served as the foundation for all subsequent NNs. Neural MT is a complete “encoder-decoder” structure that uses NN to learn the mapping between natural languages [7]. According to the hidden layer vector output by the encoder, the decoder predicts word for word to produce the word sequence of the target end. The encoder reads the source language sentences and encodes them into a set of hidden layer vector representations with fixed dimensions. Different network structures can be used to implement the MT model's encoder and decoder [8]. This has led to the successful application of deep neural networks (DNNs), such as CNN (convolutional neural network) and RNN (recurrent neural network), to the field of natural language processing. The network uses the vectorization of words or sentences as its premise and conducts feature learning [9] during training in order to learn features with higher abstraction, avoiding the need for extensive feature engineering and producing impressive results. In the most recent stage of MT development, neural MT has significantly improved its output results in terms of loyalty and fluency when compared to the conventional phrase-based MT. However, there are currently still a lot of issues with neural MT, and the level of translation still needs to be raised. On the basis of this, this essay discusses the translation of Japanese literature and ANN-based NLU. The following are its innovations:

1. In this paper, the machine automatically learns features, transforms corpus data into word vectors by distributed representation, and uses NN to realize the direct mapping between the source language and target language. At the same time, a semantic word vector construction method and a part-of-speech enhancement word vector method supervised by part-of-speech information are proposed. Through the rational use of multi-source information such as semantic knowledge base and part-of-speech sequence in NN training, the precision of word semantic expression is improved, and the performance of many natural language comprehension tasks is improved.
2. In this paper, NN parser is adopted, and “encoder-decoder” architecture based on the attention mechanism is adopted in the implementation part, which can predict the assembly sequence and parameters of modules, and has the function of automatic learning, thus improving the flexibility of the model. At the same time, the pseudoparallel corpus generated by the reverse translation method is further enhanced by low-frequency word substitution, and a grammar error correction module is additionally added in low-resource scenes to reduce grammar errors.

## 2. Related Work

MT has both theoretical value and practical value and has experienced considerable development since it was proposed. At present, the application of the DL method makes neural MT become mainstream. Nakayama et al. found that in the process of cross-domain translation, unknown words are an important factor causing translation errors. Therefore, dictionary mining technology is used for unknown word mining in domain adaptation tasks to solve the translation problem of unregistered words in new domains in domain adaptation problems [10]. Hwang presented a CNN-based framework that incorporates short text representations for classification. These representations are combined with regular conceptualized words and related concepts in a knowledge base on top of pretrained word vectors [11]. Mcshane et al. used domain knowledge to filter out domain-related bilingual parallel corpora from large-scale general data when training translation models [12]. Ni reduces the impact of unregistered words on the overall translation performance of sentences through data generalization, improves the translation quality of unregistered words themselves, and uses a multi-coverage fusion model to improve the attention scoring mechanism to further alleviate overtranslation and neural MT in neural MT (missing translation problem) [13]. Wang et al. used semantic role information to label nonterminal symbols in syntactic translation models, making translation rules more discriminative, and incorporating semantic information as a feature into existing translation models [14]. Misra proposed a CNN model that combines word and sentence features for Chinese entity relation extraction and achieved better results than existing models on the ACE2005 dataset [15]. Zhao proposed a general annotation model based on NN. For all labeling tasks, only very simple and general features are used as the input to the NN model, and word nesting is additionally introduced to initialize edge weights for the NN [16]. Jsa proposes an end-to-end modular network, which learns to generate the network structure without resorting to a parser while learning the network parameters [17]. The method proposed by Ferrari A utilizes the statistical information of massive texts and fuses it with quantified semantic knowledge to train a new semantic expression model under a unified model framework [18]. This method has achieved remarkable results on many well-known natural language understanding tasks.

However, at present, there are still many problems in neural MT, and the quality of translation still needs to be improved. Based on this, this paper focuses on the semantic expression and reasoning methods of natural language based on NN and studies the semantic expression of words, the NN model for common sense reasoning, the construction method of common sense knowledge base, and Japanese literary language translation. In this paper, NN parser is adopted, and the implementation part adopts the “encoder-decoder” architecture based on the attention mechanism, which can predict the assembly sequence and parameters of modules, and has the function of automatic learning, thus improving the flexibility of the model. At the same time, the pseudoparallel corpus generated by the reverse translation method is further enhanced by low-frequency word substitution, and a grammar error correction module is additionally added in low-resource scenes to reduce grammar errors.

## 3. Basic Principle of Artificial Nerve MT

The mathematical simulation and modeling of human brain neurons are where ANN got its start. One of the simplest and most widely applied NN models is feedforward. The fundamental elements of a multilayer feedforward network are layered, with the output of one layer's node connected to the input of the next layer's node by a forward edge. It is possible to think of the multilayer feedforward NN as a function whose input and output are both vectors. With the quick development of DL, neural MT's performance has unquestionably outperformed traditional statistical MT, and it has not only become the standard research approach for MT but also the foundational technology of for-profit online MT systems like Google and Baidu. The model structure of NN is shown in Figure 1.

According to the backbone network, MT models can be divided into the following categories: MT models based on RNN, MT models based on CNN [19], and neural MT models based on self-attention mechanism. This article will introduce them one by one.

### 3.1. MT Model Based on RNN

A recursive NN with direction can be obtained after data input in the classic DL network known as the loop NN. As a result of the signal's ability to pass through a layer indefinitely, RNN's scoring path length approaches infinity. Generally speaking, when designing NN, there should be at least three noninput layers or score paths greater than two, and a very deep layer network should have deep layers or score paths greater than ten. The deep network used in the practical design is typically a multi-level ANN with millions of free parameters and multiple hidden layers. NN propagates information using forward feedback in each iteration of the loop before using the algorithm to learn. The output of the previously hidden layer node is saved in the context node, which then uses this data to determine the state of the previously hidden layer node [20]. Traditional NN cannot handle the task of serial data prediction, but this model can. Sequence data processing is a specialty of NN. The RNN has a “memory” function because of its network properties; it will recall the input data from a previous moment and use that information to influence the output of the current moment. From the feedforward NN, the loop NN developed. A hidden layer state is also output by each layer of the loop NN, which is used when the current layer processes the following sample. Every hidden layer state at a given instant is a functional representation of every hidden layer state at the instant before. RNN only includes a limited number of return roads from the output of the hidden layer to its own input in comparison to feedforward NN. RNN can theoretically map all historical input information to the current output, whereas feedforward NN can only map the current input to the output, which seems to change little but has a significant impact on the labeling task.

### 3.2. MT Model Based on CNN

NN is a depth NN that has a convolution operation layer attached. Typically, it has a downsampling layer, two trainable nonlinear convolution layers, two full connection layers, and at least two fixed nonlinear convolution layers. This makes there at least five hidden layers. In the convolution layer, the value of the convolution kernel template is initially set at random. One objective of CNN is to train an appropriate convolution kernel, which will allow the training image to pass through and produce the desired output. Both the encoder and the decoder in the CNN-based MT model are based on CNN [21]. The main advantage of this approach is that, unlike RNN, which must be operated in a specific order, a set of data can be input into the model and calculated simultaneously. Neuron nodes between layers and adjacent layers are connected by targeted partial connections rather than full connections in the convolution process. This is done to mimic the biological NN principle, which states that only a small number of neurons in the upper layer contribute to the perception of an area by a given neuron. This connection method has many benefits, and it is because of this advancement that CNN stands out in many tasks. Equivariant representation, parameter sharing, and sparse interaction are characteristics of convolution. The number of connections and program runtime can both be significantly reduced by sparse interaction. When parameters are shared, it is not necessary to learn a unique parameter set for every position but rather just one, which can significantly reduce the number of parameters. An equation is said to be equivariant if the input changes and the result changes in the same manner. The efficiency of the MT model, which is based on CNN, is greatly increased. In a similar vein, CNN does not experience the gradient disappearance and explosion issues that RNNs do, and the number of network layers can be stacked deep using the residual connection.

The source language should be translated while taking into account all of the context information, that is, relevant at the time. NN can remember the context information and store the time sequence information by iteratively scanning the input sequence. The word vector produced by this method, however, only takes into account the left context information and does not take into account the right context information. Network models that can handle text-related tasks well include CNN and RNN. CNN retains a specific amount of text sequence information, which is equivalent to N-gram data, by setting the size of the convolution kernel, or the window value. Additionally, since a convolution operation does not require the calculation of a time sequence, multiple convolution kernels may be calculated simultaneously, improving efficiency. The MT model based on CNN has great advantages over RNN in terms of computing efficiency, but it also has its own benefits and drawbacks when it comes to extracting text sequence features. Compared to CNN, which is constrained by the convolution window size, loop NN is better able to retain the information of the entire sentence. The dependency between words should be our first point of focus because this will affect how the deep convolution network interprets the information from the entire sentence. The neural MT model typically updates the model's parameters using the gradient back propagation algorithm in order to reduce the loss function value of the model and train model parameters that can fit the data set effectively. The most widely used gradient descent algorithm is the random gradient descent algorithm.

### 3.3. Neural MT Model Based on Self-Attention Mechanism

The encoder's job is to encrypt the input's original language; the decoder, meanwhile, decodes the transmitted data that has been encoded and then creates the target language. Furthermore, you can simulate the translation process using a NN model, train the sample parameters, and learn it. When both the input and the output are variable-length sequences, the model framework can be built using an encoder-decoder, in which the encoder corresponds to the input sequence and the decoder to the output sequence. In the encoding stage, the entire source sequence is encoded into a vector, and in the decoding stage, the entire target sequence is decoded by maximizing the probability of the predicted sequence. In a neural MT model built on an encoder-decoder framework, the encoder first converts a sentence from the source language into a fixed-length semantic vector, and the decoder then uses that vector to continuously generate the target words. For translating short sentences, an encoder-decoder framework is more appropriate. It is simple to lose information when dealing with long sentences because the information vector cannot completely cover the source data. Therefore, the attention mechanism will be incorporated into the encoder-decoder framework to address this issue, and the attention mechanism will extract all coding information.  Figure 2 shows the decoder framework.

An encoder-decoder model called the transformer is made entirely of a feedforward NN and a self-attention mechanism. The position information, which is crucial for language comprehension and creation, is not taken into account by the encoder and decoder based on total attention networks, so the transformer model adds position coding to the input vectors of the lowest encoder and decoder. The attention mechanism in the decoder model improves the sequence's ability to be represented. The attention mechanism, decoder, and encoder are the three components of the neural MT model. Instead of using fixed vectors to represent the information from the source language, a collection of multiple vectors is used. The target sequence is generated using a dynamic selection of the background vector, and the decoding process concentrates on the source language portion, that is, most pertinent to the target sequence. In order to speed up computation and enhance the effectiveness of the translation model in MT, attention mechanisms are primarily used in image recognition. The transformer model has two clear benefits because of the self-attention mechanism: Parallel processing accelerates training significantly. The distance between words is 1, which more accurately depicts long-distance dependence, and the self-attention mechanism can capture global information better at 2 than it can at 1. Transformer decoder, like the encoder, has N isomorphic network layers. Each network layer has three subnetwork layers; the self-attention network is the first of these. The multi-head attention network is located at layer two. Feedforward NN with full connectivity makes up the third layer.

## 4. NN Modeling Japanese Literary Language Translation and Natural Language Understanding

Literature translation refers to the act of translating literary works in one language into another. As far as literary translation is concerned, it is not only the translation of one word into another but also the communication and collision of cultures. Japan is an implicit and tactful nation, which is not direct in language expression and likes to bend around. In contrast, China is more explicit, frank, and able to express its views directly. Therefore, in the translation of Japanese literary language, more attention should be paid to the extraction of language features. The importance of feature extraction is mainly reflected in preventing overfitting and simplifying operations on the premise of ensuring accuracy. Especially when dealing with a large amount of data. ANN is widely used in the field of natural language processing because of its autonomous learning ability of features and its ability to simplify feature engineering. Japanese literary language translation and natural language understanding are complicated. If the same network is used, the network will be large in scale, complex in structure, long in learning and application, and poor in reliability. Therefore, this paper designs the network as an integrated NN. Each sub-NN corresponds to a kind of sentence component. Samples are designed for each part, and the corresponding weights are obtained through supervised learning and stored in the form of data files. When the network works, the general control module runs the corresponding subnetwork according to the different parts of the sentence.  Figure 3 shows a neural MT model with an attention mechanism.

Let the parameter bit *w* of the NN model, given the input *x*, the probability that the NN output *x* belongs to each category *C*_*k*_ is *P*(*C*_*k*_*|x*, *w*). We can get the probabilities of all input class pairs on the training data *S*:

(1) $$\begin{array}{c} P\left(S|x\right)=\prod_{\left(x,z\right)\in S}P\left(z|x,w\right). \end{array}$$

According to the principle of maximum likelihood parameter estimation, we hope that the final parameters can make the probability distribution predicted by the model fit the data distribution in the training set as much as possible, that is, the maximization formula. From this, the maximum likelihood parameter *w*_*ML*_ can be expressed as:

(2) $$\begin{array}{c} w_{ML}=\arg\max P\left(S|w\right)=\arg\max\prod_{\left(x,z\right)\in S}P\left(z|x,w\right). \end{array}$$

In practice, the negative logarithm of *w*_*ML*_, *O* bits *P*(*S|w*) is usually obtained by minimizing the objective function *O*:

(3) $$\begin{array}{c} O=-In\prod_{\left(x,z\right)}p\left(z|x,w\right)=-\sum_{\left(x,z\right)}\text{Inp}\left(z|x,w\right). \end{array}$$

Since the logarithmic function *In* is a monotonically increasing function, minimizing −*InP*(*S|w*) is equivalent to maximizing *P*(*S|w*).

In the convolution process, the convolution kernel is used to convolve the original matrix, extract higher abstract features, and generate a new matrix. In text convolution, one dimension of convolution should be consistent with the dimension of the word vector. Therefore, only one dimension can be changed, and this dimension represents the window value. Its physical meaning is that the length of words with order relationships corresponding to each convolution operation is similar to N-gram, which can keep the relative order information within a certain length.

Suppose, *X*={*x*_1_, *x*_2_, *x*_3_,…, *x*_*T*_} represents the source language sentence sequence; *y*_*t*_ represents the output target word of the decoder at the *t* moment; *h*_*t*_ represents the output vector of the encoder at the time of *t*; *s*_*t*_ represents the hidden state of the decoder at the time of *t*; *c*_*t*_ represents the semantic vector dynamically generated by the model at the time of *t*. The dynamic generation comes from the attention mechanism, and its calculation formula is as follows:

(4) $$\begin{array}{c} c_{t}=\text{attention}\left(s_{t-1},h\;\right)=\sum_{i=1}^{T}a_{t,i}h_{i}. \end{array}$$

Among them, *a*_*t*,*i*_ represents the weight coefficient of the encoder output *h*_*t*_ at *t* time, and *a*_*t*,*i*_ satisfies the following formula:

(5) $$\begin{array}{c} \sum_{j=1}^{T}a_{t,j}=1. \end{array}$$

Equations (4) and (5) show that the essence of the attention mechanism is to obtain the weighted average, and the dynamic semantic vector *c*_*t*_ is equal to the weighted average of the output vector of *t* encoder. Among them, the calculation method of the weighting coefficient *a*_*t*,*i*_ is shown in formula (6):

(6) $$\begin{array}{c} \begin{array}{cc} a_{t,i}=\frac{\text{exp}\left(e_{t,i}\right)}{\sum_{j=1}^{T}\text{exp}\left(e_{t,j}\right)} & a_{t,i}=\frac{\exp\left(e_{t,i}\right)}{\sum_{j=1}^{T}\text{exp}\left(e_{t,j}\right)} \end{array}. \end{array}$$

Among them, *e*_*t*,*i*_ is calculated by a feedforward NN, and the abovementioned formula means that a Softmax layer is added at the tail of this feedforward NN, and the attention weight coefficient is calculated. In order to introduce vocabulary semantic knowledge, this paper proposes that the quantitative table of semantic knowledge is not semantic similarity inequality, as shown below:

(7) $$\begin{array}{c} \text{Similarity}\left(w_{i},w_{j}\right)>\text{Similarity}\left(w_{i},w_{k}\right). \end{array}$$

Among them, *w*_*i*_, *w*_*j*_, and *w*_*k*_, respectively, represent three words in the dictionary. Through semantic similarity inequality, the similar relationship between words can be effectively expressed. In the semantic vector space, semantic similarity can be further expressed in the form of formula (8):

(8) $$\begin{array}{c} \text{Sim}\left(w_{i},w_{j}\right)>\text{Sim}\left(w_{i},w_{k}\right). \end{array}$$

Where *w*_*i*_, *w*_*j*_, and *w*_*k*_ represent the semantic vectors of words *i*, *j*, and *k*, respectively.

Use a convolution kernel of length *k* for convolution, focusing on the *i* th window, then the word vector in it should have as:

(9) $$\begin{array}{c} w_{i}=v\left(x_{i}\right);v\left(x_{i+1}\right);\ldots ;v\left(x_{i+k-1}\right). \end{array}$$

After convolution, *m* vectors are obtained, *p*_1_, *p*_2_, *p*_3_,…, *p*_*m*_. Where *p*_*i*_ ∈ *R*^*d*_conv_^.

(10) $$\begin{array}{c} p_{i}=g\left(w_{i}W+b\right), \end{array}$$

where *g* is a nonlinear activation function.

Gradient descent method can easily fall into the local optimum. One solution to this problem is to introduce momentum. This method can be seen as introducing momentum or increasing inertia in the current updating direction when the weights are updated. After entering the local optimum, the weights are continuously updated under the influence of inertia, and it is possible to rush out of the local optimum. The weight updating formula after introducing momentum is as follows:

(11) $$\begin{array}{c} \Delta w\left(n\right)=m\Delta w\left(n-1\right)-a\frac{\partial O}{\partial w\left(n\right)}. \end{array}$$

Among them, 0 ≤ *m* ≤ 1 is the momentum parameter.

The process of downsampling has been streamlined. In this procedure, the convolution matrix's features are sampled using the corresponding sampling function, and the most crucial features are then extracted. This greatly reduces the matrix's dimensions and streamlines the calculation procedure while maintaining the integrity of the important features. In contrast to conventional reasoning techniques like the Bayesian network, this model uses NN as a global approximation model to directly calculate the association probability between two events instead of assuming a specific graph structure. Without relying on preexisting artificial knowledge, this mechanism will enable the model in this paper to train and learn from samples effectively. The idea of the attention mechanism is that by retaining the intermediate output results of the encoder on the input sequence, the decoder at different times will pay attention to different input parts, and the output at each time has its own semantic vector *C*_*i*_. The alignment network between the source language sequence and the target language sequence is actually established by the introduction of the attention mechanism. The initial fixed length and invariant semantic vector will change into a dynamic semantic vector matrix after the attention mechanism weighting. Long sentences can now be represented much more effectively. In other words, the translation effect of the translation model for long sentences has significantly improved as compared to the model without the attention mechanism as a result of the introduction of the attention mechanism. The trained ANN translation model is employed in this study as the foundational transfer learning model. Retrain the deep parameters of the Japanese literary language using transfer learning to extract its characteristics and enhance the MT model's capacity for learning. Additionally, unlike the conventional graph model, the event dependency structure diagram will not need to be designed in advance for this paper, greatly enhancing the model's adaptability and generalizability.

## 5. Result Analysis and Discussion

In order to achieve better experimental results, the translation model is trained in the hardware environment of GPU processing acceleration, which is TeslaM60. The machine learning framework is Transformer, and the script language is python. The low-frequency word replacement module needs to obtain the position of the word to be replaced in the target language through the alignment model, so it is necessary to use the existing parallel corpus to train the alignment model in advance. The alignment model adopts fast_align tool. The grammar error correction module generates a large number of sentences with grammatical errors by adding noise and combines them with real sentences to form training data so that the grammar error correction module can be trained. Set warmup_steps in this chapter to 4000. In order to prevent overfitting in training, a dropout mechanism is introduced. When decoding, the beam search algorithm is used and a length penalty is introduced to choose a better translation result. The word embedding size is set to 512, the number of network layers is set to 6, the batch size is set to 2048, the learning rate is set to 0.9, the number of iterations is set to 2000 rounds, and the dropout value is set to 0.1. In this paper, the data are normalized. The normalization of the verification set and test set uses the mean and standard deviation obtained from the training set. The normalization of input data has a significant impact on the experimental results in our experiments, so the input data are normalized by default in all experiments in this paper. Due to the small sample data, the translation effect of MT model is often poor. In order to achieve better results, after processing the word vectors by Word2vec, a small neural translation model is trained first, and then the neural MT model is trained on a large scale by using transfer learning technology. ReLU is used as an activation function and Adam is used as an optimizer in model training. Adam optimizer will dynamically adjust the learning rate during training. Firstly, set the warm_step, and the learning rate will increase linearly within the warm_step. After warm_step, the learning rate will gradually decline. The dimension of the input layer word nesting is fixed to 100. The dimension of the output layer is determined by the specific task and is the number of categories that the task needs to mark. Similarity values range from 0 to 10, and the increase in numerical value represents the increase in word similarity. In this task, to measure the performance of the semantic expression model, in fact, we use the trained semantic word vectors to score the similarity of word pairs in the test set and analyze the correlation between the scoring results and the manually marked scores.

The quality of training data directly affects the performance of the neural MT model. In order to better train the MT model, firstly, the Word2vec model is used to preprocess Japanese, and then the one-dimensional continuous vector is obtained through Word2Vec mapping, and then the trained word vector is used in MT model training. When training, the validation set is used to determine whether to stop training. If the model for 10 rounds in a row does not get better performance in the validation set, the training is terminated, and the model with the best performance on the validation set is used for testing. The data preprocessing step includes: filtering sentences with sequence lengths over 50 in the original corpus; Filter sentences with the length ratio of the source language to target language exceeding 1.5. Use the trained BPE tool to segment the corpus, and add <bos> and <eos> markers at the beginning and end. After preprocessing, the training corpus totals 2,692,541 sentence pairs. The data set is shown in Table 1.

In order to evaluate the experimental results more objectively, BLEU will be used as the evaluation index in the experiment. BLEU is an estimation based on the similarity between system output and manual reference translation. If the value of BLEU is higher, it means that the similarity of translation results is higher, the translation effect is better, and the model performance is superior.  Figure 4 shows the comparison results of different training methods.

It can be seen that the training speed of this method is slightly faster than that of the comparison method. It is found that the model proposed in this paper can cluster words according to their part of speech. On this level, this model can improve the expressive ability of semantic models. In order to further verify this assumption, this paper conducts unsupervised part-of-speech clustering operations on words according to their semantic expression vectors. The results are shown in Figure 5.

At the same time, in order to verify the effect of adding attention mechanism NN translation network model, this experiment compares the training speed and model performance of the traditional NN model and RNN model with this model. The comparison results are shown in Figure 6.

As can be seen from Figure 6, the training convergence rate of NN translation model with the attention mechanism is obviously faster. The model with attention mechanism has better performance and better effect on Japanese literary language translation and natural language understanding.  Figure 7 shows the relationship between corpus size and corresponding BLEU in different scenarios.

Figure 7 serves as additional evidence of the neural MT's reliance on data. Whether it is a low-resource scenario or a scenario with abundant resources, the BLEU value on the test set also increases as the scale of training data does. The pseudobilingual corpus created by the artificial data enhancement method has limited performance improvement for translation tasks, and its growth cannot continue indefinitely. This is because the BLEU increasing trend gradually slows down. The experiment will use BLEU to assess the translation of various models into the Japanese literary language in order to verify the translation effect of the MT model after migration. This paper adopts the same experimental configuration, including the use of training algorithms and fundamental linguistic features, which are consistent with it, in order to achieve a fair comparative experiment. The evaluation results are shown in Table 2.

It can be seen intuitively from the data in the table that the BLEU value of the model proposed in this paper is higher. This shows that the translation quality of the proposed model is higher. After training through transfer learning, the translation effect of Japanese literary language has been significantly improved. After translating the generalization part, it is necessary to replace the generalization marker in the translation with the translation result. In the process of generalization, similar generalized components in the same sentence have been labeled with serial numbers, so there is no need to consider the alignment of similar generalized components in the same sentence when replacing, and the final translation result can be obtained by direct replacement. The accuracy of different models in Japanese literary language translation is shown in Figure 8.

It can be seen that the accuracy of this algorithm can reach about 95%. In order to further verify the experimental results, based on the data set of this chapter, this paper compares the translation accuracy of Japanese literary language between this model and the traditional model. The comparison results obtained are shown in Table 3.

It can be seen from the comparison results in the table that the recall rate and F value of this model for Japanese literary language translation are higher than those of the comparison model. It can be concluded that this model has a good effect on Japanese literary language translation and natural language understanding, and can realize the accurate translation of Japanese literary language.

## 6. Conclusion

Literary works not only express some thoughts and connotations of the author but also reflect the culture of a country. Based on ANN, this paper discusses the translation of Japanese literary language and the understanding of natural language. In this paper, NN parser is adopted, and the implementation part adopts the “encoder-decoder” architecture based on the attention mechanism, which can predict the assembly sequence and parameters of modules, and has the function of automatic learning, thus improving the flexibility of the model. At the same time, a semantic word vector construction method and a part-of-speech enhancement word vector method supervised by part-of-speech information are proposed. Through the rational use of multi-source information such as semantic knowledge base and part-of-speech sequence in NN training, the precision of word semantic expression is improved, and the performance of many natural language comprehension tasks is improved. Simulation results show that the accuracy of this algorithm can reach about 95%, and the recall rate can reach about 96%. After adding language features and transfer learning to NNMT, the training speed of MT model can be improved. This method effectively solves the problem of information loss and greatly improves the flexibility and popularization of the model. It can provide some reference for literary language translation and natural language understanding. In the next step, we can try to use the cluster to run the network model, which can save time and cost, and also run more complex networks.

## Figures and Tables

**Figure 1:** NN model structure.

**Figure 2:** Decoder framework.

**Figure 3:** Add the neural MT model of attention mechanism.

**Figure 4:** Comparison of results of different training methods.

**Figure 5:** Comparison of clustering effect of the model.

**Figure 6:** Performance comparison of different models.

**Figure 7:** The relationship between corpus size and BLEU value change.

**Figure 8:** Accuracy of different models in Japanese literary language translation.

**Table 1:** Dataset information.

Type		Name	Size
Parallel corpus	Training set	WMT2016EN-DE	4.1 M
	Verification set	Newstest	8K
	Test set	Newstest	4K

Monolingual corpus		News crawl corpus	WMT2015EN-DE

**Table 2:** Translation evaluation results of different translation models.

Model	Japanese	Chinese
RNN model	0.19	0.25
Convolution model	0.21	0.26
Model of this paper	0.34	0.36

**Table 3:** Performance comparison of different translation models.

Model	Recall rate (%)	F Value (%)
RNN model	82.39	84.57
Convolution model	85.96	87.41
Language feature model	86.71	84.79
Model of this paper	89.42	92.46

## Data Availability

The data used to support the findings of this study can be obtained from the author upon request.
